This article has been retracted.

# Difference between Acyclovir and Ganciclovir in the Treatment of Children with Epstein–Barr Virus-Associated Infectious Mononucleosis

**DOI:** 10.1155/2021/8996934

**Published:** 2021-10-20

**Authors:** Shouyuan Zhang, Yanyan Zhu, Yanyan Jin, Hong Sun, Weiqun Wang, Lu Zhan

**Affiliations:** ^1^Department of Pediatrics, Zhejiang Hospital of Integrated Traditional Chinese and Western Medicine, Hangzhou, Zhejiang 310003, China; ^2^Department of Pediatrics, Hangzhou Children's Hospital, Hangzhou, Zhejiang 310010, China; ^3^Department of Pediatrics, Children's Hospital Affiliated to Zhejiang University, Hangzhou, Zhejiang 310003, China

## Abstract

**Objective:**

To investigate the efficacy differences between acyclovir and ganciclovir in the treatment of children with Epstein–Barr virus (EBV)- associated infectious mononucleosis (IM).

**Methods:**

A total of 128 children with EBV-IM who were admitted to our hospital from February 2019 to February 2021 were selected and randomly divided into the acyclovir group (*n* = 64) and the ganciclovir group (*n* = 64) according to the random number table method. All the children were given symptomatic treatments such as protecting the liver and reducing fever. On this basis, the acyclovir group was given an intravenous drip of acyclovir, while the ganciclovir group was given an intravenous drip of ganciclovir. The treatment was continued for 7 days. After the treatment, the clinical efficacy, disappearance time of symptoms and signs, related blood routine indexes, EBV-DNA negative conversion rate, and the incidence of adverse reactions during the treatment were compared between the two groups.

**Results:**

After treatment, the total effective rate of the ganciclovir group (92.19%) was higher than that of the acyclovir group (73.44%) and the difference was statistically significant (*P* < 0.05). The disappearance time for the symptoms and signs of angina, fever, lymphadenopathy, hepatomegaly, and splenomegaly in the ganciclovir group was lower than that in the acyclovir group, and the difference was statistically significant (*P* < 0.05). After treatment, the levels of atypical lymphocyte proportion, lymphocyte proportion, and WBC count in the two groups were lower than those before treatment, the levels in the ganciclovir group were lower than those in the acyclovir group, and the difference was statistically significant (*P* < 0.05). After treatment, the EBV-DNA negative conversion rate (81.25%) in the ganciclovir group was higher than that in the acyclovir group (60.93%) and the difference was statistically significant (*P* < 0.05). During treatment, the incidence of adverse reactions in the ganciclovir group was significantly lower than that in the acyclovir group and the difference was statistically significant (*P* < 0.05).

**Conclusion:**

In the treatment of children with EBV-IM, the therapeutic effect of ganciclovir is obviously superior to that of acyclovir. Ganciclovir can quickly eliminate the symptoms of angina, fever, enlarged lymph nodes, and other signs in children, can improve abnormal blood indicators, and has a higher negative conversion rate of EBV and less adverse reactions.

## 1. Introduction

Infectious mononucleosis (IM) has a high incidence rate in children, which is often caused by the infection by the herpes family virus Epstein–Barr virus (EBV). The main clinical symptoms include angina, fever, hepatosplenomegaly, and so on [1]. If not treated in time, the disease easily develops into a malignant disease related to chronic active EBV infection and causes multisystem damage [2]. Compared with adults, it is more harmful in children. In addition to symptomatic treatment, the use of antiviral drugs for the treatment of EBV-IM has been widely recognized in clinical practice; however, the optimal choice of antiviral drugs is still controversial [3]. Acyclovir and ganciclovir are nucleoside broad-spectrum antiviral drugs, and acyclovir is mainly used for herpes virus infections, such as herpes zoster and chicken pox [4, 5]. Ganciclovir is mainly used for cytomegalovirus infection, and it is widely used in AIDS patients and patients undergoing chemotherapy for cancer [6]. Acyclovir and ganciclovir have been used to some extent in the treatment of diseases associated with EB virus infection, while acyclovir is more common and works better than other antiviral drugs [7]. However, differences in the efficacy and safety of acyclovir and ganciclovir in the treatment of EBV-IM in children are rarely reported. Therefore, this study explored and compared the efficacy and safety differences between acyclovir and ganciclovir in the treatment of EBV-IM in children. Specific reports are provided in the following sections.

## 2. Materials and Methods

### 2.1. Research Objects

A total of 128 children with EBV-IM who were admitted to our hospital from February 2019 to February 2021 were selected and randomly divided into the acyclovir group (*n* = 64) and the ganciclovir group (*n* = 64) according to the random number table method. Inclusion criteria were as follows: children who met the diagnostic criteria of IM, with typical symptoms such as fever, angina, and lymphadenopathy, with the proportion of atypical lymphocytes >10% and increase in the proportion of lymphocytes and white blood cell (WBC) counts; with EBV-DNA test positive; who were between the ages of 1 and 12 years; with good compliance. Exclusion criteria were as follows: allergy to acyclovir or ganciclovir; severe immune dysfunction; severe organ dysfunction. The acyclovir group included 32 males and 30 females. Their age ranged from 1 to 9 years, with an average of (4.68 ± 2.11) years. The course of disease ranged from 2 to 14 days, with an average course of (6.33 ± 2.35) days. The ganciclovir group included 33 males and 29 females. Their age ranged from 1 to 9 years, with an average of (4.59 ± 2.153) years. The course of disease ranged from 2 to 14 days, with an average course of (6.82 ± 2.52) days. There was no significant difference in general information between the two groups (*P* < 0.05). This study was approved by the Ethics Committee of our hospital.

### 2.2. Research Methods

#### 2.2.1. Therapeutic Method

All children were given symptomatic treatments such as liver protection and myocardial nutrition support. On this basis, the acyclovir group was given acyclovir injection (10 mg/kg) combined with 100 ml glucose injection using an intravenous drip twice a day. The ganciclovir group was given ganciclovir injection (10 mg/kg) combined with 100 ml glucose injection using an intravenous drip twice a day. All patients were treated with a slow drip, and each drip lasted more than 1 hour. All children were treated continuously for 7 days, during which the drug dose was adjusted according to the adverse reactions and remission degree of the disease. (In order to avoid the interference of different drug injection methods on the experimental results, acyclovir and ganciclovir were slowly and intravenously injected in the same way in this study.)

#### 2.2.2. Observation Index

The disappearance time of typical IM symptoms of the two groups of children was recorded and compared, including angina, fever, lymphadenopathy, hepatomegaly, and splenomegaly.

Before and after treatment, all children were given routine blood tests. Atypical lymphocyte ratio, lymphocyte ratio, and leukocyte count were compared between the two groups.

Before and after treatment, the fluorescence quantitative polymerase chain reaction (PCR) test was used to detect the EBV-DNA level in the whole blood of children. The number of cycle times (CT value) required for the fluorescence intensity of the sample to reach the threshold value was ≤ 39, representing the positivity of EBV-DNA in children. The negative conversion rates, decline, and no changes (including increases) were compared between the two groups.

The adverse reactions including arrhythmia, abnormal liver function, thrombocytopenia, leukopenia, and gastrointestinal reaction were recorded and compared between the two groups during the treatment. (If the child suffers from new liver dysfunction during treatment or the liver dysfunction aggravates, the liver dysfunction will be considered as an adverse reaction of the therapeutic drugs.)

#### 2.2.3. Efficacy Criteria

Markedly effective criteria are as follows: within 3 days after medication, the temperature returns to normal within 3 days, EBV-DNA becomes negative or decrease, and clinical symptoms such as angina and hepatosplenomegaly significantly improve or disappear. Effective criteria are as follows: within 5 days after medication, the temperature returns to normal, EBV-DNA decreases, and clinical symptoms such as angina and hepatosplenomegaly improve or disappear. Unless otherwise stated above, it shall be deemed as invalid. Total effective rate = (markedly effective cases + effective cases)/total cases × 100%.

### 2.3. Statistical Methods

SPSS19.0 software was used for processing, measurement data were expressed by mean ± standard deviation (mean ± SD), and pairwise comparison was analyzed by the *t*-test. The enumeration data were compared among groups using the *χ2* test. *P* < 0.05 indicates that the difference was statistically significant.

## 3. Results

### 3.1. Comparison of Clinical Effects between Two Groups

After treatment, the total effective rate of the ganciclovir group (92.19%) was higher than that of the acyclovir group (73.44%) and the difference was statistically significant (*P* < 0.05), as shown in Table 1.

### 3.2. Comparison of Disappearance Time of Clinical Symptoms and Physical Signs between Two Groups

The disappearance time for the symptoms and signs of angina, fever, lymphadenopathy, hepatomegaly, and splenomegaly in the ganciclovir group was lower than that in the acyclovir group and the difference was statistically significant (*P* < 0.05), as shown in Figure 1.

### 3.3. Comparison of Related Blood Routine Indexes between Two Groups

After treatment, the levels of atypical lymphocyte proportion, lymphocyte proportion, and WBC count in the two groups were lower than those before treatment, the levels in the ganciclovir group were lower than those in the acyclovir group, and the difference was statistically significant (*P* < 0.05), as shown in Figures 2∼4.

### 3.4. Comparison of EBV-DNA Negative Conversion Rate between Two Groups

After treatment, the EBV-DNA negative conversion rate (81.25%) in the ganciclovir group was higher than that in the acyclovir group (60.93%) and the difference was statistically significant (*P* < 0.05), as shown in Table 2.

### 3.5. Comparison of the Incidence of Adverse Reactions between Two Groups

During treatment, the incidence of adverse reactions in the ganciclovir group was significantly lower than that in the acyclovir group and the difference was statistically significant (*P* < 0.05), as shown in Table 3.

## 4. Discussion

Children's IM is mostly caused by EBV, which is one of the herpes viruses. EBV can cause damages to multiple organs of the whole body and can be transmitted through the respiratory tract [8]. When IM is caused, the clinical manifestations mainly include sore throat, fever, lymph nodes, hepatosplenomegaly, and so on. When the disease is at the beginning stage, the routine blood test is usually unremarkable, so EBV has a high rate of being missed and misdiagnosed. If it is not treated in time, the disease can develop rapidly and even lead to disability or death [9, 10]. At present, there is no specific drug for the treatment of IM and symptomatic treatment is often adopted to enhance the autoimmune function of children, and antiviral drug intervention is combined to significantly improve the treatment effect. Clinically, many drugs are used against EBV, such as acyclovir, ganciclovir, and ribavirin. Ganciclovir is a derivative of acyclovir. They are nucleoside antiviral drugs that have the function of inhibiting the synthesis of EBV-DNA. The anti-EBV effect of them is stronger than other drugs [11, 12]. However, the therapeutic effect and difference between them in the treatment of children with EBV-IM are still uncertain.

The results of this study showed that after treatment, the total effective rate of the ganciclovir group was significantly higher than that of the acyclovir group and the disappearance time of typical clinical symptoms such as angina, fever, and hepatosplenomegaly in the ganciclovir group was significantly lower than that in the acyclovir group. Acyclovir and ganciclovir both showed good effects on abnormally high proportion of abnormal lymphocytes, proportion of lymphocytes, and white blood cell count, but ganciclovir showed better effects. Ganciclovir has a broader antiviral spectrum than acyclovir, and the DNA polymerase of the EBV is highly sensitive to both triphosphates of acyclovir and ganciclovir [13, 14]. Ganciclovir is converted into activated triphosphate by thymidine kinase action in infected cells, which competitively inhibits viral DNA polymerase, terminates EBV-DNA prolongation, and inhibits replication of its viral products. Furthermore, ganciclovir is more water soluble than acyclovir, and the drug activity of ganciclovir in Epstein–Barr virus infected cells is 100 times higher than that in non-Epstein–Barr virus infected cells, where its efficacy can last for several days. Acyclovir does not have these characteristics, so ganciclovir has better curative effect [15].

EBV infection can cause hemophagocytic syndrome, myocarditis, lymphoma, meningitis, and many other critical illnesses, and children's immune system is not yet fully developed, so their condition develops more rapidly [16]. With the increase in the EBV-DNA load, the risk of complications, the degree of organ damage, the severity of the disease, and the mortality rate of children are significantly increased [17]. In children whose symptoms have resolved but in whom EBV is still not positive, there is still a certain risk of recurrent episodes of IM that develop into chronic EB virus infection [18]. The quantitative PCR test can accurately reflect the degree of EBV infection and the number of virus replications in children. EBV-DNA test results showed that after seven days of treatment, the negative conversion rate of EBV-DNA in the ganciclovir group was 81.25%, significantly higher than that of the acyclovir group (60.93%). In addition, only 6 children in the ganciclovir group had the same viral load, while 12 children in the acyclovir group had the same viral load. However, it was possible that because of the small sample size, the comparison between the two groups of unchanged children was not statistically significant. The above results indicated that ganciclovir had a stronger antiviral effect against EB virus than acyclovir. Hence, timely application of ganciclovir to children with IM could effectively prevent a series of other critical illnesses caused by EB virus, such as meningitis, in children.

Although acyclovir and ganciclovir have good effects on the treatment of EBV-IM, they have certain cytotoxicity, which can cause liver and kidney damage, thrombocytopenia, gastrointestinal dysfunction, and other adverse reactions [19]. Therefore, clinicians are more cautious in their application to child patients. Studies have shown that intravenous infusion of ganciclovir and other drugs can achieve good curative effect, but it will also lead to an increase in adverse reactions [20]. In order to reduce the possible adverse reactions in children, all children in this study were treated with slow intravenous infusion (the infusion time was more than 1 hour). The treatment results showed that under the same dose and infusion method, the incidence rates of adverse reactions such as arrhythmia, liver dysfunction, and thrombocytopenia in the ganciclovir group were lower than those in the acyclovir group and the safety rate of ganciclovir was higher.

## 5. Conclusion

In the treatment of EBV-IM, the therapeutic effect of ganciclovir is obviously superior to that of acyclovir. Ganciclovir can quickly eliminate the symptoms of angina, fever, enlarged lymph nodes, and other signs in children, can improve abnormal blood indicators, and has a higher negative conversion rate of EBV and less adverse reactions.

## Figures and Tables

**Figure 1:** Comparison of disappearance time of clinical symptoms and physical signs between two groups. Note: compared with the acyclovir group, ^*∗*^*P* < 0.05.

**Figure 2:** Comparison of the atypical lymphocyte proportion between two groups. Note: compared with the acyclovir group, ^*∗*^*P* < 0.05.

**Figure 3:** Comparison of the lymphocyte proportion between two groups. Note: compared with the acyclovir group, ^*∗*^*P* < 0.05.

**Figure 4:** Comparison of the WBC count between two groups. Note: compared with the acyclovir group, ^*∗*^*P* < 0.05.

**Table 1:** Comparison of clinical effects between two groups (*n*, %).

Groups	Markedly effective	Effective	Ineffective	Total effective rate
Acyclovir group (*n* = 64)	16	31	17	47 (73.44)
Ganciclovir group (*n* = 64)	26	33	5	59 (92.19)
*χ* ^2^ value				7.904
*P* value				0.005

**Table 2:** Comparison of EBV-DNA negative conversion rate between two groups (*n*, %).

Groups	Negative	Decline	No change
Acyclovir group (*n* = 64)	39 (60.93%)	13	12
Ganciclovir group (*n* = 64)	52 (81.25%)	16	6
*χ* ^2^ value	6.424	0.401	2.327
*P* value	0.011	0.526	0.127

**Table 3:** Comparison of the incidence of adverse reactions between two groups (*n*, %).

Groups	Arrhythmia	Abnormal liver function	Thrombocytopenia	Leukopenia	Gastrointestinal disorder	Total adverse reactions
Acyclovir group (*n* = 64)	5	1	2	3	4	15 (23.44)
Ganciclovir group (*n* = 64)	0	0	1	1	3	5 (7.81)
*χ* ^2^ value						5.926
*P* value						0.015

## Data Availability

The data used and/or analyzed during the current study are available from the corresponding author upon request.
